# The Effect of Shenyi Capsule on Non-Small-Cell Lung Cancer Combined with Chemotherapy from the *Yin-Yang* Perspective

**DOI:** 10.1155/2021/1653750

**Published:** 2021-08-18

**Authors:** Zhixing Cai, Yue Teng, Yue Chen

**Affiliations:** ^1^Department of T.C.M, Tongren Hospital, Shanghai Jiao Tong University School of Medicine, 1111 Xianxia Road, Shanghai 200336, China; ^2^Outpatient Department of Clinic Center, Yueyang Hospital of Integrated Traditional Chinese and Western Medicine, Shanghai University of Traditional Chinese Medicine, 110 Ganhe Road, Shanghai 200437, China

## Abstract

As an example of Shenyi capsule on non-small-cell lung cancer combined with chemotherapy, this review discusses the synergistic effect and mechanism of natural drugs in oncotherapy from the *yin-yang* perspective in ancient Chinese philosophy, so as to reflect the therapeutic principle of natural drugs for tumor more comprehensively. The major focuses of this review are on the philosophical thinking of *yin-yang* as a tool which can not only explain the effect of Shenyi capsule in NSCLC combined with chemotherapy but also explore the mechanism of Shenyi capsule at the cellular and molecular level. Learning from the “*yin-yang*” thinking of ancient Chinese philosophy will bring more enlightenment to the research and development of traditional Chinese drugs in the future.

## 1. Introduction

Ginseng, a natural plant medicine, has been used in Asia for thousands of years [1]. Ginsenoside Rg3 in ginseng has been proved to have potential antitumor activity against a variety of malignant tumors [2]. Shenyi capsule, a kind of new single Chinese medicine highly purified by ginsenoside Rg3 based on modern pharmaceutical technology, was included in NCCN (2016) and has been widely used in the treatment of non-small-cell lung cancer (NSCLC) combined with chemotherapy.

However, existing studies have found that [3–5], through the metabolic transformation, the Rg3 monomer still needs to be transformed into 20(s) ginsenoside Rg3 and other isomers in order to play an antitumor role (Figures 1(a)–1(c)). Research on the mechanism of Rg3 has also found that the antitumor effect of Rg3 has been actually realized through multiple levels of gene, protein, and pathway expression [6–9]. How to collect the antitumor mechanism information of Rg3 and comprehensively evaluate [10] the effect of Shenyi capsule plus chemotherapy on advanced NSCLC has always been a major bottleneck in the study of combined treatment.

Yin-yang in ancient Chinese philosophy describes the close, complementary, and subtle relationship between two opposites. Yin-yang theory, which originated from ancient Chinese philosophy, was introduced into traditional Chinese medicine (TCM) by Huangdi's Internal Classic [11]. The theory treats diseases from the perspective of “integration” and attaches importance to the role of “yin-yang balance” in the treatment. Such an ancient Chinese philosophical thinking is increasingly being used for reference and introduced into the treatment of major diseases such as malignant tumors [12–14].

This paper attempts to use the yin-yang thinking of ancient Chinese philosophy to discuss the role of Shenyi capsule on NSCLC combined with chemotherapy, in order to provide a more comprehensive way to interpret the effect and mechanism of natural herbal drugs in oncotherapy.

## 2. *Yin-Yang* Attribute of Shenyi Capsule

According to the original text of Shennong's Herbal Classic, “ginseng can nourish the five zang organs and prolong the life.” In the long-term practice, TCM doctors have concluded that ginseng has the effect of “invigorating vital energy, replenishing qi, and promoting body fluids.” In the TCM field, the effect of “invigorating energy” belongs to “yang,” while that of “generating body fluids” pertains to “yin.” Therefore, ginseng itself has the characteristics of yin-yang coexistence. As a monomer extract of ginseng, Shenyi capsule has the same attribute, that is, “yin-yang coexistence.”

Existing studies have confirmed that ginsenoside Rg3 [15] can significantly improve the weight of immune organs (spleen and thymus), lymphocyte transformation ability, and NK cell activity of tumor-bearing mice and improve nonspecific and specific (including cellular and humoral) immune functions of mice [16], which coincides with the “tonifying” effect of ginseng. Moreover, related studies have shown that Shenyi capsule can inhibit proliferation [17], induce apoptosis [18–20], and inhibit invasion and metastasis [21, 22] and other direct cytotoxic effects in the same direction as traditional chemotherapeutic drugs by enhancing the inhibition of the PI3K/AKT/mTOR signaling pathway [23]. Meanwhile, unlike traditional chemotherapeutics, Shenyi capsule can also inhibit tumor neovascularization [24] and prevent it from spreading, promote the maturity of residual tumor vessels, and restore the homeostasis of its structure and function, thus effectively inhibiting tumor by changing the local microenvironment [25].

Therefore, from the perspective of tumor inhibition mechanism, Shenyi capsule not only includes “positive reconstruction” of the immune system based on the whole body but also contains “negative inhibition” of local tumors. It not only has the same “direct tumor inhibition” effect as traditional chemotherapy but also has the repair effect of the “tumor vascular microenvironment” which is different from traditional chemotherapy. This multilevel antitumor mechanism constitutes the “antitumor” network of Shenyi capsule, and it is difficult to explain the network's whole picture with microscopic cytobiology. However, traditional Chinese philosophy can help us better understand the essence of antitumor effect of Shenyi capsule combined with chemotherapy. It holds that all the objective laws of nature belong to yin-yang, which determines the nature of all things; that is, the so-called “one yin and one yang is called Tao” (the Book of Change·Xi Ci I), “Out of Tao, one is born; out of one, two; out of two, three; and out of three, the created universe“(the Book of Tao and Teh). Such a simple expression, however, can help us better understand the interdependence and close interaction between “the whole and parts,” “the negative tumor inhibition, and positive immunity” between Shenyi capsule and NSCLC chemotherapy.

## 3. *Yin-Yang* Balance Effect of Shenyi Capsule

The first meta-analysis of chemotherapy and optimal supportive treatment for advanced NSCLC published in the Journal of Clinical Oncology (2008) has confirmed that supportive treatment combined with chemotherapy can improve the survival rate of advanced NSCLC [26, 27] and has a significant effect in reducing toxic side effects [28] and chemoresistance [29] of chemotherapy. Obviously, chemotherapy has a direct cytotoxic effect on NSCLC [30–32], while Shenyi capsule synergically increases the efficacy of chemotherapy by reducing toxicity, increasing sensitization, enhancing immunity, etc. They are obviously opposite, interdependent, and complementary to each other, that is, the so-called “yin-yang relationship.” In the view of ancient Chinese philosophy, “yin and yang are the compendium of all things” (Huangdi's Internal Classic·Great Theory on Yin-Yang Corresponding to Nature). Yin-yang is the general principle of all; drawing lessons from such a principle, we have found that Shenyi capsule and chemotherapy can also be ascribed to “yin-yang.” Specifically, Shenyi capsule can be classified as “yang,” which is always in opposite directions of chemotherapy's “yin” in terms of chemoresistance and dose-effect toxicity; thus, Shenyi capsule has always been playing a regulatory role of “balancing”(Huangdi's Internal Classic·Discussion on Decoction and Wine) in the treatment of NSCLC combined with chemotherapy.

### 3.1. Attenuation-Sensitization Effects of Shenyi Capsule

#### 3.1.1. Toxic Side Effects and Chemoresistance of Chemotherapy

Platinum-based chemotherapy is currently the first-line treatment for advanced NSCLC [33]. Almost all platinum preparations have serious toxic side effects such as digestive reaction and bone marrow suppression [34]. Chemoresistance is a basic problem that limits the efficacy of many chemotherapy regimens [35]. In recent years, we have tried to avoid toxic side effects and chemoresistance as much as possible through drug combination [34–37]. Because there is no single mechanism that can explain the nature of toxic side effects and chemoresistance, the combination therapy based on different mechanisms cannot really get rid of them.

Aiming at the abovementioned defects of chemotherapy, the combination of Shenyi capsule mainly improves severe acute vomiting above Grade II [27] and effectively improves hemocytotoxicity and platelet inhibition caused by chemotherapy [27]. Due to the “vascular inhibition effect” of Shenyi capsule [38], the “vascular network” that tumors depend on for survival is blocked, and the rapid proliferation of tumor during the intermittent period of chemotherapeutics is also blocked, which effectively consolidates the phased curative effect achieved by chemotherapy. Meanwhile, this “vascular normalization” [39] overcomes the barrier of chemotherapeutic drugs entering tumor cells and enables more chemotherapeutic drugs to contact tumor cells, so as to play a direct cytotoxic role, thus improving the chemosensitivity of NSCLC.

If we refer to “yin-yang,” it is not difficult to find that the toxic side effects and chemoresistance, like the efficacy of chemotherapy, is actually the other side of it and the two sides coexist closely (Figure 2). If there are no toxic side effects and chemoresistance, there will be no curative effect of chemotherapy at all, that is, the “mutual rooting of yin and yang” (Jingyue Book·Chuanzhong Lu·Yin-yang). Therefore, the toxic side effects and chemoresistance are inevitable by either the new regimen of dual chemotherapy [40] or the new route of oral chemotherapeutic medication [41].

On the contrary, the synergistic and sensitized pathway of Shenyi capsule does not target any known mechanism of producing toxic side effects and chemoresistance [42–44]. Instead, it ultimately changes the “abnormal” nature of tumor by transforming the relationship of the tumor vascular network, reflecting Chinese philosophical thinking of “relationship determines nature” [45]. Thus, it skillfully bypasses the inevitable problem of toxic side effects and chemoresistance and achieves the purpose of reducing toxicity and increasing sensitization in synergistic chemotherapy.

### 3.2. Shenyi Capsule's Dose-Effect Synergy

#### 3.2.1. Chemotherapeutics' Dose-Effect Toxicity

As mentioned above, platinum-based chemotherapeutic agents have significant cytotoxicity. With the progression of NSCLC, there will be a problem, that is, “time/course-dose toxicity-”related cytotoxic accumulation [46]. In order to consider the pharmacological and toxicological safety, the maximum dose of chemotherapeutic agents for NSCLC intervention must be strictly set. Moreover, in order to restore the myelosuppressive toxicity, intermittent treatment with conventional chemotherapeutic agents is indispensable, which creates an opportunity for cancerous cells to proliferate and rebound. According to the principle of tumor growth dynamics [47], tumor cell proliferation will be more active in the intermittent period of chemotherapeutics, which also hinders the efficacy of NSCLC chemotherapy.

Compared with platinum-based drugs, Rg3 has a “time/course-dose effect-”related antitumor effect on NSCLC [48–50]. Due to the “vascular inhibition effect” of Shenyi capsule [51], the “vascular network” that tumors depend on for survival is blocked, and the rapid proliferation of tumors in the intermittent period of chemotherapeutics is also blocked, thus effectively consolidating the phased treatment achievements and improving the curative efficacy of chemotherapy. It has been observed that, with the progress of NSCLC treatment, the “toxicity” of chemotherapeutics has gradually become prominent, showing the characteristic of impeding “curative effect” and limiting the dosage of chemotherapeutics to a certain extent. This kind of interaction between “toxicity and efficacy” can catalyze the change of the dominant position due to certain conditions, which is similar to the concept of “yin-yang growth and decline ” in ancient Chinese philosophy. “Yin and yang are intermixed, resulting in a change” (Huangdi's Internal Classic·Great Theory on Law of Primordial Qi in Nature), so the purpose of combined medication is to prevent the “change in the extreme phase” between “chemotoxicity and efficacy” [52] and to achieve “yin-yang balance” between the maximum of curative effect and the optimization of combined dose (Figures 3(a)-3(b)).

## 4. *Yang Generates Yin Waxes* Mechanism of Shenyi Capsule

As mentioned above, Shenyi capsule can play the “same direction” cytotoxic effect with chemotherapeutic medication, similar to the concept of “mutual rooting of yin and yang” in ancient Chinese philosophy, namely, “yang grows yin waxes” (Huangdi's Internal Classic·Plain Conversation·Great Theory on Yin-Yang Corresponding to Nature). According to the currently known synergistic mechanism, the interdependent and mutually promoting “yin-yang interaction” between Shenyi capsule and chemotherapy in the course of NSCLC treatment will be described one by one (Figure 4).

### 4.1. Enhancing the Inhibition Rate of Cell Proliferation

Platinum-based drugs exert cytotoxic effects by inhibiting DNA replication and transcription in lung cancer cells [53]. Different from platinum-based drugs with an aperiodic specific broad-spectrum cytotoxic effect, ginsenoside Rg3, the main active ingredient of Shenyi capsule, plays a cytotoxic role by preventing the proliferation cycle of G2/M cancer cells [54]. Studies have shown that [55] Rg3 combined with chemotherapy can significantly enhance the expression of cyclin B, D1, and *E*, as well as cyclin dependent kinases 2 and 4, leading to growth block of tumor cells in the G0/G1 phase. It can be seen that the combination therapy of “yang generates while yin waxes” can enhance the inhibition rate of tumor cell proliferation through the superposition of (non) cyclic-specific cytotoxic effects.

### 4.2. Activating Apoptosis Factors

The caspases family plays an important role in cell apoptosis [56]. Bcl-2 family proteins are key regulatory factors in the process of cell apoptosis [56]. Overexpression of Bcl-2 antiapoptotic proteins [56] can prevent cell apoptosis, ultimately causing tumor. NF-*κ*B activation [57] and IAP protein expression [58] also play important roles in the regulation of cancerous cell apoptosis. Research findings have shown that [9, 59–61] compared with chemotherapy alone, Rg3 combined with chemotherapy can significantly enhance the expression of caspase-3/8 and caspase-9, inhibit the overexpression of Bcl-2, and significantly inhibit the expression of IAP protein (IAP-1) and x-chromosome IAP (XIAP). The ratio of Bax/Bcl-2 was significantly increased by inhibiting the activation of NF-*κ*B. Another combination therapy of Rg3 and cisplatin has shown that [62] the combination regimen of “yang waxes yin wanes” not only reduces Bcl-2 expression but also activates endogenous apoptotic pathways.

### 4.3. Regulating Cell Invasion and Metastasis

Inhibiting cell invasion and metastasis is an effective way of antitumor therapy. Ginsenoside Rg3, the main active component of Shenyi capsule, inhibits tumor migration by inhibiting [61] proto-oncogene (C-Myc), cyclooxygenase-2 (COX-2), and matrix metalloproteinase-9 (MMP-9). Rg3 combined with chemotherapy, exactly as the mutual restriction of yin and yang, can [63] not only downregulate the expression of EMT-related factors but also upregulate that of E-cadherin protein, so as to regulate cell invasion and metastasis.

### 4.4. Boosting Neovascularization Inhibition

Inhibition of tumor angiogenesis [64], by restraining tumor-induced angiogenesis, depriving the tumor of its necessary blood supply and resulting in the stagnation of tumor expansion, is one of the effective means of tumor inhibition. Compared with chemotherapy alone, Rg3 combined with chemotherapy [65] can not only inhibit tumor neovascularization but also moderately antagonize the generated ones; in addition, it can reduce the expression of VEGF and Bcl-2 and cut down microvessel density of the target tissue. Multiple studies have shown that [65, 66] continuous low doses (1/10–1/3 of the maximum tolerated dose) of certain cellular toxicants can improve chemotherapy efficacy by targeting tumor microvessels. This so-called “antitumor angiogenesis” chemotherapy regimen not only blocks tumor angiogenesis, which is the “yin” of tangible substance, but also restrains the disorder expansion of tumor, which is the “yang” of intangible way, thus providing a new approach to NSCLC treatment.

### 4.5. Promoting Positive Immune Drift

Immune surveillance under physiological state can identify and control new tumor cells. In the pathological state where immune surveillance is dysfunctional or even lost, tumor immunosuppression, immune tolerance, and immune escape mediated by multiple mechanisms promote tumor progression [67]. Targeted therapy for patients with immune mutant genes [68–70] significantly improves the efficacy of advanced tumors. However, the proportion of these genomic changes among NSCLC patients is small and eventually produces acquired drug resistance due to secondary gene mutations; therefore, chemotherapy is still needed [71].

At present, it has been confirmed that [72], with the progress of advanced NSCLC, the ratio of FOXP3+/CD8+ in NSCLC tissues increases, and the infiltration of Treg cells in the microenvironment of noncancerous NSCLC tissues increases significantly. Shenyi capsule can [73–75] promote the proliferation of lymphocytes and make CD3+, CD4+, lymphocytes, and Th1/Th2 drift to the positive immune direction, thus ameliorating the immune function. The combination of Shenyi capsule and chemotherapy [76] can increase the proportion of NK+, CD3+, and CD4+ cells to a greater extent and reduce the percentage of CD8+ cells, in order to regulate the immune function of NSCLC via bidirectional adjustment in terms of CD8+/CD4+.

## 5. Discussion

### 5.1. *Yin Wanes Yang Waxes* Effect of Shenyi Capsule

As mentioned in Huangdi's Internal Classic·Plain Conversation·Great Theory on Yin-Yang Corresponding to Nature, “yang transforms qi while yin shapes into configuration.” It can be seen that the formation of NSCLC is consistent with the process of “yin's shaping into configuration” [53, 61, 65, 66]. In addition, the internal accumulation problems such as “dose-effect toxicity” of chemical drugs can also be seen as “yin's shaping into configuration,” while the immune regulation effect of Shenyi capsule is similar to that of “yang transforms qi” described in Huangdi's Internal Classic [72–76]. The combination of chemical drugs and Shenyi capsule, on the one hand, plays the role of “yin” of chemotherapy in inhibiting tumors and, on the other hand, plays the role of “yang” of Shenyi capsule in enhancing the immune function; moreover, it reduces the “yin” of chemotherapeutic toxic side effects from the perspective of “positive immunity.” Therefore, the curative effect of Shenyi capsule on NSCLC combined with chemotherapy is a reflection of the synergistic effect of TCM, which is “*yin wanes while yang waxes*.”

### 5.2. *Strengthening Yang Suppressing Yin* Advantage of Shenyi Capsule

As mentioned above, Shenyi capsule, on the one hand, plays the role of “yin” in inhibiting tumors by “antitumor angiogenesis” and, on the other hand, plays the role of “yang” in promoting immune regulation by “positive immune drift.” Different from traditional chemical drugs, the two-way regulation of “strengthening yang and suppressing yin” is mostly realized through the transformation of the blood supply network [39], immune monitoring [67], and other tumor microenvironment of NSCLC. Therefore, the body immunity itself is retained to the maximum extent, and the tolerance of the body to chemical drugs is improved as well. Consequently, in the treatment of NSCLC, the combination of Shenyi capsule and chemical drugs has a better clinical advantage than chemotherapy alone [27].

### 5.3. Yin-Yang Philosophical Significance of Shenyi Capsule

This paper discusses the effect and mechanism of Shenyi capsule on NSCLC combined with chemotherapy. It is not difficult to find that, different from the direct “negative inhibition” of chemotherapy, Shenyi capsule always exerts a “positive promotion” effect of synergistic chemotherapy. Under the subdivision, this “positive promotion” includes not only “positive-negative” bidirectional regulation of Shenyi capsule on chemotherapy efficacy [77–79], toxic side effects, and chemoresistance [80, 81] but also “positive immune” regulation of the combined therapy [76]. Further subdivided, we can find from the mechanism level that Shenyi capsule, which is different from the “direct antitumor” cytotoxic effect of chemotherapy drugs, mainly achieves indirect antitumor effect by inhibiting the “vascular” network, on which NSCLC depends for survival. If we continue to subdivide the molecular biological mechanism of Shenyi capsule in the combined chemotherapy, some findings would be explored from the microscopic “signal pathway,” “protein,” “gene,” and other multiple levels.

In fact, the occurrence and development of NSCLC has always been existed, and with the help of medical science and technology, the understanding of cancer is continuously deepening. However, this progressive cognitive level has been described by “yin-yang” thinking of TCM for thousands of years. “The scope of yin-yang in heaven and earth is so extensive that, after further deduction in the specific application, it can be deduced from ten to one hundred, from one hundred to one thousand, from one thousand to ten thousand, and even innumerable. However, the general principle is still no more than the yin-yang principle, that is, unity of opposites“(Huangdi's Internal Classic·Plain Conversation·On Separation and Combination of Yin and Yang). “Unity” is the holistic concept of TCM, with yin-yang as a whole, it can be divided into innumerable parts of yin and yang, and such parts can be integrated into the whole. Therefore, Shenyi capsule, combined with chemotherapy, regulates the local lung tissue lesions from the holistic yin-yang perspective, which is the concrete embodiment of the “concept of holism” of TCM, and also achieves the actual curative effect superior to chemotherapy alone.

## 6. Conclusions

In this paper, taking Shenyi capsule combined with chemotherapy on NSCLC as an example, we have tried to evaluate the effect of natural drugs in oncotherapy from the yin-yang perspective, so as to reflect the treatment principle of natural drugs in oncotherapy more comprehensively [47]. It has been proved that the philosophical thinking of “yin-yang” can not only appropriately explain the “attenuation,” “sensitization,” and “synergistic” effects of combined therapy but also fully explore the “gene-protein-pathway” mechanism found at the “micro” cellular and molecular level. Therefore, we believe that referring to “yin-yang” thinking of traditional philosophy will bring more enlightenment to the research and development of traditional Chinese drugs; moreover, its possible mechanism of action will be explored more comprehensively (Figure 5).

## Figures and Tables

**Figure 1:** (a) Ginsenoside Rg3. (b) 20(S) ginsenoside Rg3. (c) 20(R) ginsenoside Rg3.

**Figure 2:** Diagram of “intermixed rooting of yin and yang.”

**Figure 3:** (a) Chemotherapy presents a periodic “yin-yang crisscross” (*y* = COSx) before treatment. (b) The combination therapy of Shenyi capsule and chemotherapeutic drugs alone present the same direction of periodic attenuation and synergistic effect.

**Figure 4:** “Yang generates yin waxes” mechanism of Shenyi capsule in NSCLC chemotherapy.

**Figure 5:** Antitumor mechanism and immune regulation of Shenyi capsule from the yin-yang perspective.

## Abbreviations

NSCLC: Non-small-cell lung cancer
NCCN: National Comprehensive Cancer Network
NK cell: Natural killer cell
PI3K: Phosphatidylinositol 3-kinase
AKT: Protein kinase B
mTOR: Mammalian target of rapamycin
DNA: Deoxyribonucleic acid
G2/M: Second gap/metaphase
G0/*G*1: Stop phase /first gap
Bcl-2: B-cell lymphoma/leukemia-2 protein
Bax: Bcl-2-associated X protein
IAP: Inhibitor apoptosis protein
XIAP: X-linked inhibitor apoptosis protein
NF-*κ*B: Nuclear factor kappa-B
C-Myc: Cancer-myc
COX-2: Cyclooxygenase-2
MMP-9: Matrix metalloproteinase 9
EMT: Epithelial mesenchymal transformation
VEGF: Vascular endothelial growth factor
FOXP3: Forkhead box P3
CD8: CD8-positive T-lymphocytes
CD4: CD4-positive T-lymphocytes
TCM: Traditional Chinese medicine.
